The article "Sports Rehabilitation Treatment of Medical Information in Tertiary Hospitals Based on Computer Machine Learning" was retracted in 2023. Reasons: signs of a paper mill; compromised peer review; unreliable results or conclusions.

# Sports Rehabilitation Treatment of Medical Information in Tertiary Hospitals Based on Computer Machine Learning

**DOI:** 10.1155/2022/4219976

**Published:** 2022-06-25

**Authors:** Xiaojun Ma, Zhenfeng Zhang

**Affiliations:** ^1^School of Physical Education, South China University of Technology, Guangzhou 510640, Guangdong, China; ^2^Zhenzhou University of Aeronautics, Zhenzhou 450046, Hena, China

## Abstract

**Objective:**

The processing and analysis of medical rehabilitation information data in tertiary hospitals is a hot research topic. Combining medical data analysis with machine learning algorithms to improve data mining efficiency is a problem that needs to be solved at present. This paper proposes an autonomous perception model of sports medicine rehabilitation equipment based on a deep learning algorithm for sports medical rehabilitation data.

**Methods:**

This paper cites a deep learning multi-dimensional perception model for medical rehabilitation equipment autonomous perception. The model utilizes the automatic overhaul of medical rehabilitation equipment based on deep belief networks. This paper extracts features through a multi-layer neural network and obtains fault location results of medical rehabilitation equipment through softmax.

**Results:**

In similarity prediction, the accuracy rate of the first three kinds of feedback containing the target answer is 77%. The accuracy rate of the target answers included in the top five kinds of feedback was 92%.

**Conclusion:**

In this study, it is feasible to apply deep learning to the quality control information system of sports rehabilitation medical equipment. This improves the management efficiency of medical rehabilitation equipment to a certain extent.

## 1. Introduction

The medical equipment purchased and used by many tertiary hospitals is generally under the responsibility of the equipment department. The daily maintenance and management of this medical equipment mainly include the perception of its status in the medical equipment software system and the integration of data, self-judgment of equipment failure, and evaluation of equipment failure. The active early warning of faults also includes the equipment's identification of its faults and the automatic generation of relevant information. From the beginning of use to the scrapping of medical equipment, the medical equipment software system's perception of itself and the early warning of possible failures are significant [1]. The software system is of great significance to the smooth operation of the medical equipment during its use, the elimination of faults, and the perception of its state. Equipment fault diagnosis and early warning have multi-dimensional support. The operation and maintenance process of sizeable medical equipment includes unstructured and structured data structures of faults generated during use. The data generated by different medical equipment have multiple sources and different data frame structures, which can utilize multi-source heterogeneity. Building a principal system of big data sharing among medical equipment provides an example of the different data generated by different medical equipment in large and medium-sized medical institutions. Relevant personnel need to build a self-perception model of multi-source heterogeneous data generated between different medical devices and provide automatic early warning for perception results. This is essential work in intelligent medical equipment.

## 2. Model Architecture Design

The specific architecture of the system is shown in Figure 1. The multi-dimensional operation and maintenance status perception layer of medical equipment adopts sensor cluster collection. This provides the underlying data for fault awareness [2]. Unstructured medical equipment multi-source heterogeneous fault data are unstructured for the underlying data. This forms a pool of failure data samples available for machine learning applications. The intelligent perception and active early warning layer of medical equipment failures introduce machine learning multi-dimensional perception. It plays the role of iteratively updating the mapping relationship between fault perception and active warning. The active early warning mechanism for medical equipment failures constructed by it realizes the self-evolution of the fault-tolerant performance of medical equipment. The visual human-computer interaction layer realizes friendly human-computer interaction under cross platform through dynamic visual technology. The logic diagram of the control flow of the medical equipment operation and maintenance status autonomous perception and active early warning model is shown in Figure 2.

### 2.1. Monitoring Module

The monitoring module collects the voltage, current, temperature and humidity, logs, and other internal operating status data of various medical equipment in real time by integrating different sensors and processors [3]. It transmits data for subsequent work via a built-in IoT card. At the same time, the power supply of the monitoring module is provided through USB.

### 2.2. Transmission Module

The monitoring module transmits the collected operating status data of the medical equipment to the data analysis module through the built-in IoT card. At this time, we can set the transmission timing to ensure the timeliness of data collection and transmission.

### 2.3. Analysis and Maintenance Module

We use big data, an expert knowledge base, and other technologies to perform data mining and analysis on these parameters according to the received real-time status data of the equipment. This article judges whether the diagnostic equipment is regular by comparing the normal parameters of the equipment [4]. We assess the current state of a component and predict future trends. The stand-alone comparison refers to establishing a benchmark model based on the historical data of the device's health status through machine self-learning and other methods. When monitoring equipment parameters that have unhealthy trends, it will be reminded.

### 2.4. Model Realization and Simulation Verification

#### 2.4.1. Sub-Model of Autonomous Perception of Medical Equipment Operation and Maintenance Status

We use the Puhws-how open-source dataset for large-scale equipment state awareness to construct an unstructured multi-source heterogeneous fault data sample pool for medical equipment [5]. In this paper, the policy network *m* is used as an actor based on the complex and variable parameters of the medical equipment state data carrier and the multi-source heterogeneity. This paper uses a value network to fit the (*s*, *a*) function of playing the critic's role. The evaluation function of the pros and cons of the self-awareness strategy *m* of the multi-dimensional operation and maintenance state of medical equipment under the situation of dynamic topology change is as follows:

(1) $$\begin{array}{c} L\left(s,a|\theta \right)=E_{s,a,r,s^{\prime }}\left[{\left(Q^{*}\left(s,a|\theta \right)-y\right)}^{2},{\left(Q^{*}\left(s,a|\theta \right)+y\right)}^{2}\right]. \end{array}$$

Based on (1), this paper gives the deterministic strategy formula of multiple *Q* network structures. Because the multiple *Q* network structure adopts a random strategy, to obtain the current action, it is necessary to sample the probability distribution of the optimal strategy [6]. The entire action space is integrated at each step in the iterative process. This paper adopts a deterministic strategy based on the target *Q* network. In this paper, the perception strategy is determined directly through the function according to the behaviour. *m* in the formula is generally understood as an optimal behaviour strategy *a*_*t*_=*μ*(*s*_*t*_*|*1 − *θ*^*μ*^), and the optimal function for the distributed perception of multi-source heterogeneous data can be characterized as follows:

(2) $$\begin{array}{c} J\left(\mu_{\theta }\right)=\int_{S_{s}}^{S_{e}}\rho^{\mu }\left(s\right)\mu_{\theta }\left(s\right)\text{d}s\\ =E_{s∼\rho^{\mu }}\left[r\left(s,\mu_{\theta }\left(s\right)\right)\right]. \end{array}$$

Equation (2) is unstable in the big data flow environment. In this paper, the first-order derivation processing of formula (2) is performed, and the optimal generation mechanism of the multiple *Q* network structure can be expressed as formula (3). It has strong compatibility. We can better realize the autonomous perception and memory of significant data-level multi-source heterogeneous procurement constraints.

(3) $$\begin{array}{c} \nabla_{\theta }J\left(\mu_{\theta }\right)=\int_{S_{s}}^{S_{e}}\rho^{\mu }\left(s\right)\nabla_{\theta }\mu_{\theta }\left(s\right)Q^{\mu }\left(s,a\right){|}_{a=\mu_{\theta }}ds=E_{s∼\rho^{\mu }}\left[\mu_{\theta }\left(s\right)Q^{\mu }\left(s,a\right){|}_{a=\mu_{\theta }}\right]. \end{array}$$

#### 2.4.2. Sub-Model of Active Early Warning of Medical Equipment Failure

We use policy network *μ* to act as *actor* according to the complex and variable multi-source and heterogeneous characteristics of medical equipment's multi-dimensional operation and maintenance parameters. We use a value network to fit the (*s*, *a*) function to play the role of *critic*. This paper will integrate the early warning objective function of the deep deterministic policy gradient algorithm with the empirical buffer factor:

(4) $$\begin{array}{c} J\left(\theta^{\mu }\right)=E_{\theta^{\mu }}\left[r_{1}+\gamma r_{2}+\gamma^{2}r_{3}+\cdots \right]. \end{array}$$

The *Q* function is expressed as the reward expectation for choosing an action under a deterministic policy *μ*. In this paper, the empirical buffer factor is introduced in the coupling link between the policy network and the *Q* network. At this time, the iterative convergence speed of the algorithm is improved by orders of magnitude. We randomly sample mini-batch data from a pool of empirical buffer factors. Since different sub-policies will be executed in different rounds, we can get a memory replay pool for each training round. Finally, we solve the fusion objective function's gradient for each training round's sub-policy parameters [7]. At this point, we can autonomously identify the fault information frame and mark it. The active warning trigger function is represented by the following formula:

(5) $$\begin{array}{c} \nabla_{\theta_{i}}J\approx \frac{1}{S}\sum_{j}\nabla_{\theta_{i}}\mu_{i}{\left(o_{i}^{j}\right)\nabla_{a_{i}}Q_{i}^{\mu }\left(x^{j},a_{1}^{j},\ldots ,a_{i},\ldots a_{N}^{j}\right)|}_{a_{i}=\mu_{i}\left(o_{i}^{j}\right)}. \end{array}$$

The parameter *θ*^*Q*^ in the multiple *Q* networks has better self-evolution performance. In this paper, the expected return value is obtained by selecting an action in the *s* state by using the *μ* strategy with the help of *Q*^*μ*^(*s*, *μ*(*s*)). At this time, the feature framework of autonomously constructing fault information can better realize autonomous and active early warning of fault information of large-scale multi-source heterogeneous operation and maintenance data [8].

#### 2.4.3. Simulation Verification under the Typical Environment of the Model

This paper uses the data text of the operation and maintenance status of medical equipment recorded in the hospital equipment department from the second quarter of 2019 to the second quarter of 2020 as the initial training data. In this paper, based on the PyTorch open-source framework, the model is simulated and verified in the GymTorcs environment. In this paper, the algorithm is simulated and verified from the simulation diagram of the autonomous perception performance of the model's operation and maintenance state under the multi-source heterogeneous operation and maintenance data and the simulation diagram of the model's operational early warning performance under the control of the deep reinforcement learning algorithm. At the same time, this paper conducts graphical schematic simulation in Keras2.2.2 and Gym0.10.8 environments [9]. We use significant difference markers to give a comparison curve in the simulation graph. The final simulation results are shown in Figures 3 and 4.

#### 2.4.4. Model Engineering Application Performance Verification

This paper constructs an autonomous perception and active early warning mechanism of medical equipment operation and maintenance status with engineering application significance, as shown in Figure 5. We selected the People's Hospital equipment department as the model efficacy verification carrier. This paper uses the comprehensive management and control system for the operation and maintenance status of medical equipment, which is currently mainstream in medical institutions, as a comparison system [10]. This paper analyzes the autonomous perception and active status of medical equipment operation and maintenance from equipment status awareness coverage, data processing strategy efficiency, equipment fault discovery cycle efficiency, model active early warning accuracy, model engineering application friendliness, and early warning information push convenience. Comprehensive performance of early warning model details are shown in Table 1. In this paper, it can be concluded from the qualitative and quantitative analysis in Table 1 that the model can better realize the autonomous perception and active early warning of the operation and maintenance status of medical equipment. It has obvious advantages in terms of comprehensive perception of operation and maintenance status information, strong compatibility of medical equipment, and high efficiency of active early warning. The research results of this paper have positive significance for further promoting the implementation of competent medical care.

## 3. Conclusion

This paper uses the TensorFlow open-source training platform to verify model performance simulation in the PyCharm integrated development environment. At the same time, this paper analyzes the engineering application of the model with the equipment department of the People's Hospital as the model effectiveness verification carrier. The system can better realize real-time perception and early warning of large-scale multi-source heterogeneous fault data.

## Figures and Tables

**Figure 1:** Schematic diagram of the system architecture of medical equipment operation and maintenance status autonomous perception and active early warning model.

**Figure 2:** Logic diagram of the control flow of medical equipment operation and maintenance status autonomous perception and active early warning model.

**Figure 3:** Simulation diagram of model operation and maintenance status autonomous perception performance under multi-source heterogeneous operation and maintenance data.

**Figure 4:** Simulation diagram of the operational early warning performance of the model under the control of the deep reinforcement learning algorithm.

**Figure 5:** Schematic diagram of model engineering application performance verification layout.

**Table 1:** Comparison of engineering application efficiency of autonomous perception and active early warning models.

Project	Active duty system	Model of this paper
Device status awareness coverage (%)	76.49	93.93
The efficiency of data processing strategy (%)	68.6	91.29
Equipment fault perception accuracy (%)	74.29	90.47
Model active warning accuracy rate (%)	67.03	94.85
Model engineering application friendliness	Better	Very good
The convenience of early warning information push	General	Very good

## Data Availability

The data used to support the findings of this study are available from the corresponding author upon request.
